# Medicinal Applications of Banana Peel Flour Used as a Substitute for Computing Dietary Fiber for Wheat Flour in the Biscuit Industry

This article has been retracted.

**DOI:** 10.1155/2022/2973153

**Published:** 2022-04-22

**Authors:** Garsa Ali Alshehry

**Affiliations:** Food Science and Nutrition Department, College Science-Taif University, Saudi Arabia

## Abstract

The aim of this study, medicinal applications of banana peel flour, was used to estimate nutrition value and minerals content. The results indicated that banana peel flour was safe for food application, and it was lower in protein and fat and higher in dietary fiber and total carbohydrate which were 52.68 and 67.25%, respectively. Moreover, the minerals content of phosphorous, potassium, sodium, manganese, and calcium were 217.92, 110.24, 96.43, 85.25, and 80.27 mg/100 g, respectively. Furthermore, the problem of the study investigated the effect of banana peel flour incorporation with wheat flour with 72% extraction to produce biscuit blends at different ratios of 5.0, 10.0, 15.0, and 20.0%, respectively. The nutrition value and mineral content of banana peel flour in biscuits increased gradually in the blends, according to the results. The methods of study of the four biscuit blends were prepared with banana peel flour substituted and wheat flour extraction of 72 percent, and they were compared to a control biscuit. Sensory properties reported that the control biscuit was the highest score followed by blends which had contained 5, 10, and 15% banana peel flour. Meanwhile, the blend of biscuit fortified with 20% was not accepted by panelists. From the color biscuits, the blends containing 5, 10, and 15% banana peel flour had acceptable color, and the blends' color was not acceptable. This may be caused by dark color and high dietary fiber. The texture profile analyzer and physical characteristics were confirmed and gave the same results. The result is that it could be recommended that the banana peel flour, which has high fiber content, produce acceptable biscuits fortified with 5, 10, and 15% and become functional foods. Panelists did not find the 20% blend biscuits to be particularly appealing.

## 1. Introduction

Recovering fruit and vegetable waste into foods enhances the sustainability of the diet system. The transformation of horticultural waste into value-added ingredients and food products could lead to better human nutrition and food security [1].

Due to rising consumer interest in vitamins, minerals, unsaturated fatty acids, bioactive compounds, and fiber in food, there has been a boom in consumer interest in these nutrients in recent years. The focus is on consumer health and functional food products' wellbeing. Banana waste is repurposed. As a result, peeling could increase raw material yield.

The banana contained three genera (*Musa*, *Musella*, and *Ensete*) belonging to the Musaceae family. In addition, *Musa acuminata* and *Musella balbisiana* are the edible bananas [2, 3]. Medicinal applications of banana peel products are getting greater attention from food manufacturers by transforming them into functional food. When medicinal applications of banana peel are discarded after harvesting, they are also not usually utilized in food production [4] pointing out that the production of food products from by-products can become better for the nutritional value of them. [5] are benefitted in getting great into the utilization of by-products like a banana peel. It is a great medicinal application of banana peel containing high amounts of various nutrients that have been used to produce massive food products. The fruit processing industry is characterized by an elevated rate of waste production. Many by-products like peel, stalk, seeds, and crushed pulp still contain great amounts of bioactive compounds which are nutritional waste [6]. Banana peel contains 40% of bananas. Meanwhile, this can be converted by-product to reduce waste and create a new food source like medicinal application wastes containing high amounts of protein, fiber, and minerals. As well, it has great water and oil holding capacity; thus, it has a low-calorie product from a low-cost [7]. Moreover, [17, 18] suggested eating foods that are low in fat and calories, in addition to containing high amounts of antioxidants and dietary fiber, due to their ability to lower cholesterol and soft feces, as well as chronic heart disease disease.

In a large prospective study in the United States of America (USA), the consumption of dietary fiber was identified as a protective factor for the risk of total or cause-specific death due to various chronic diseases such as cancer, cardiovascular diseases, and diabetes mellitus, among others [8]. The reason for this is that high fiber intake improves serum lipoprotein values, reduces blood pressure, aids weight reduction, and promotes regularity [9]. There is evidence showing that soluble fibers play a part in blood glucose attenuation, cholesterol reduction, and insoluble fibers promoting laxation [10].

In addition to its nutritional benefits, the flour from banana varieties can possibly be used to produce ready-to-eat products that offer a high to combine bioactive compounds that are missing nutrients in these products [11, 12]. Next, by-products that contained great content of dietary fiber can be utilized in different industries, where they can change the compositional characteristics and elevated shelf life for different products [13]. Bananas are easily available and their low-cost processing into flour; therefore, it was used as an alternative to wheat flour [14].

Therefore, this study aims to estimate the nutritional values of banana peel as a by-product and, moreover, evaluate the quality of wheat flour and banana peel flour at different addition to produce biscuits determining chemical nutrition, color, texture analysis, and acceptability for consumers.

## 2. Materials and Methods

### 2.1. Materials

Banana, wheat flour with 72% extraction, ingredient of biscuits, and reagent-grade chemicals and food-grade polythene were obtained from the local market at Taif region, Kingdom of Saudi Arabia.

Male albino mice were used to study acute oral toxicity, and eighteen mice weighing 20–30 g were obtained from the Pharmacy College at King Saud University. Mice were housed and fed on a basal diet according to [15].

## 3. Methods

### 3.1. Preparation of Banana Peel Flour (BPF)

Bananas (*Musa sapientum*) have been washed in clean water to remove other undesirables. The bananas were peeled with the skins cut into small slices. Then, the slices were evaporated to destroy the enzymes presented and dried at 65°C for 8 hours. After that, it was cooled to room temperature and ground to obtain fine flour. Banana flour is stored in plastic bags to decompose and support biscuits.

### 3.2. Acute Oral Toxicity Test

Mice were divided into three groups of six mice each. The first group was given distilled water. The second and third groups were given the banana peel flour 2.0 and 5.0 g dissolved separately in 100 mL distilled water and taken orally at 1 mL/kg body weight/day. Animals were kept under observation for two weeks. After that, all mice were subjected to autopsy, and the mean body weight gain was calculated and compared to the control group [16].

### 3.3. Determination of Chemical Composition of Banana Peel Flour

Proximate composition of raw banana peel flour was determined by moisture, and protein, fat, crude fiber, ash, and carbohydrate were obtained by the difference according to [17].

Minerals content was determined in the banana peel flour using the atomic absorption spectrophotometer (3300 Perkin Elmer) according to [18].

### 3.4. Preparation of Biscuits Substituted with Banana Peel Flour

The four blends of biscuits were prepared from banana peel flour substituted with wheat flour with 72% extraction, and it was compared with the control biscuit. The control biscuit was made from wheat flour with 72% extraction. The first, second, third, and fourth blends contained 5, 10, 15, and 20% banana peel flour, substituted from wheat flour.

The different blends were mixed with ingredient of biscuits separately and combined well to produce appropriate dough. It was cut and then cooked for 10 to 15 min at 180 to 210°C and left to cool before being packaged in plastic bags according to [19].

### 3.5. Determination of the Nutritional Composition of Different Blends of Biscuits

Chemical composition, total dietary fiber (TDF), and its fractions and minerals content were determined in different blends of biscuits according to the above previous method.

### 3.6. Sensory Evaluation

Different blends of biscuits were evaluated for their sensory properties for twenty panelists' staff from the Food Science and Nutrition Department, College Science-Taif University, Kingdom of Saudi Arabia. Different blends of biscuits were evaluated for color, appearance, flavor, taste, texture, and overall acceptability by a nine-point Hedonic scale according to [20].

### 3.7. Color of Different Blends of Biscuits

The different blends of biscuits measured the color with a Hunter Lab Colorimeter (MiniScan XE Plus, Reston, VA) according to [21]. The color values were recorded as *L*∗, *a*∗, and *b*∗.

### 3.8. Texture Profile Analyzer of Biscuits

Different blends of biscuits were determined using a texture profile analyzer (TPA) according to [22].

### 3.9. Physical Characteristics of Biscuits

Biscuits were measured for high (mm), diameter (mm), and spread ratio according to [23]. Spread ratio = diameter/high.

### 3.10. Statistical Analysis

The findings were presented for analysis of variance; Duncan's multiple tests at the (*p* 0.05) were utilized to compare the means. The analysis was achieved by utilizing the ANOVA procedure for the statistical analysis system [24].

## 4. Results and Discussion

### 4.1. Oral Toxicity Assay

From the oral toxicity assay result from banana peel flour, it showed that all tested mice appeared normal and no mortality occurred for two weeks. There were no considerable variations for the body weight gain in all mice; the autopsy showed no significant pathological changes between treated mice and control mice. These results confirmed that the banana peel was indicating its safety for food application.

### 4.2. Chemical Composition and Minerals Content of Banana Peel Flour

Chemical analysis, total dietary, soluble, and insoluble dietary and, in addition, minerals content were determined in banana peel flour, and the results in Table 1 showed that the banana peel flour lower in protein and fat were 6.83 and 4.01% and higher crude fiber and total carbohydrate were 12.38 and 67.25%, respectively. These results confirmed with [25] who found protein, fat, and carbohydrates contents, and the banana peel flour were 5.9 g/100 g, 3.6 g/100 g, and 76.3 g/100 g, respectively. Moreover, [26] the banana peel contained more fat content than citrus peels which had 2.6 g/100 g [27].

Dietary, soluble, and insoluble dietary fiber from banana peel flour in this study were 52.68, 10.39, and 42.29 g/100d dry weight, respectively. Other studies have reported even higher values for dietary fiber content in banana peel flour, reaching 55.5% [28, 29]. The differences may be explained by fruit variety and stage of maturation and other factors such as processing methods and parameters used [30].

Moreover, the minerals content in banana peel flour with high amounts of phosphorous, potassium, sodium, manganese, and calcium were 217.92, 110.24, 96.43, 85.25, and 80.27 mg/100 g, respectively. [31] found that the banana peel is a good source of potassium, phosphorus, calcium, magnesium, and manganese, as well as the banana peel contains high phosphorus, iron, calcium, magnesium, and sodium which were 211.30, 47.00, 59.10, 44.50, and 115.10 mg/100 g, while zinc, copper, potassium, and manganese were low in content by 0.033, 0.51, 4.39, and 0.702 mg/100 g [32].

Each value represents the mean ± SD.

### 4.3. Chemical Constituents and Dietary Fiber in Different Blends of Biscuits

Chemical analysis and total dietary fiber, as well as soluble and insoluble, were determined in biscuits with different blends, and the results in Table 2 illustrated that the moisture was lower from control biscuits made from wheat flour (72% extraction) by 9.12% to 8.40% in a blend that contained 20% banana peel flour. This decreased moisture may be due to the banana peel flour lowering moisture. Biscuits with lower moisture will be free of damage and of harmful microbes and will maintain the shelf life of biscuits. Moreover, the biscuit fortified with 20% banana peel flour was the lowest in protein (8.65%), which may be because banana peel flour lowered protein.

The increase in the fat content of the different blends when the level of banana peel flour increases is due to a high-fat content in the banana peel flour [26]. The carbohydrate content of biscuits mixed with banana peel flour was considerably lower than the control biscuits. The control biscuit exhibited the highest carbohydrate content (64.70%), while 20% of banana peel flour (57.70%) had the lowest. This is due to lowering in other compositions. These results were confirmed by [11] who found that by adding defatted coconut flour which had a source of fiber, the total carbohydrates were decreased in the biscuits due to the various amounts of the chemical constituents in the defatted coconut flour.

Total dietary, soluble, and insoluble dietary fiber contents in different blends of biscuits are given in the same table. The total dietary fiber content was considerably greater with the increase in the different blends of biscuit, and the banana peel flour can be used as a substitute. The value of the total dietary fiber content in the biscuits ranged between 3.65 and 14.19%. Insoluble and soluble dietary fibers were the dominant fiber fraction in all biscuit blends. Soluble fiber is recognized to reduce cholesterol and help lower the risk of colon cancer; in addition, insoluble fiber showed the benefits of regulating the bowels and increasing stool volume. [30].

### 4.4. Minerals Content in Different Blends of Biscuit

Minerals content were determined in different blends of biscuits, and the results in Table 3 indicating calcium, sodium, potassium, phosphorus, and manganese were higher in biscuits made from 20% banana peel flour which were 89.35, 78.33, 78.29, 57.38, and 34.29 mg/100 g dry weight, respectively. Meanwhile, control biscuits were made from 72% wheat flour, which had low mineral content, and also, the different blends were gradually increased when the banana peel flour was increased. These results increased gradually when adding banana peel flour to produce different blends. With a 72% extraction, the biscuits caused the banana peel to have the highest mineral content than the wheat flour. It can be clarified that the minerals content in banana peel flour is large enough and thus has a high ash ratio. This may be due to the greatest fiber content in banana peel flour [34]. Dietary deficiency of micronutrients, like calcium and potassium, is closely related to the development of chronic heart disorders [35].

Potassium's high concentration in the banana peel can assist in maintaining blood pressure and balancing bodily fluids, as well as controlling kidney failure, cardiac difficulties, and respiratory difficulties. Because iron transports oxygen to cells, it is required for energy production, collagen formation, and the normal functioning of the immune system. Manganese aids in the development of skeletal and cartilage tissue [4].

### 4.5. Sensory Evaluation of Biscuits

The sensory properties were determined in the control biscuit and its blends, and the results in Table 4 and Figure 1 which showed the highest score for color were observed in control biscuits (9.00). As well as a significant difference with experimental biscuits of 20% banana peel flour (6.25), experimental biscuits 5, 10, and 15% were 8.25, 7.50, and 7.00, respectively. The mean texture of control and experimental biscuits ranged from 9.50 to 9.00, and the mean score of flavor ranged from 7.00 to 9.00. The addition of banana peel flour did not affect the texture and aroma scores of biscuits until 15% banana flour. The mean score of taste ranged from 6.00 to 9.00. The control biscuits (9.00) tasted the best as compared with the different blends of biscuits. Moreover, it was observed that the appearance score of biscuit was 9.00 in the control sample than the different blends which were 8.50, 7.75, 7.50, and 6.75, respectively. The mean score of overall acceptability ranged from 9.00 to 6.50. This means that the control biscuit was the highest score followed by blends which contain 5, 10, and 15% banana peel flour. Moreover, it showed a significant difference between the blend biscuit fortified with 20% banana peel flour and other different blends of biscuits.

This may be due to high protein in the flour which has contained high gluten. Contrary, the utilization of flour containing low protein will give crispy biscuits. This confirmed that good flour for making biscuits is wheat flour which contains low protein [34].

### 4.6. Color in Different Blends of Biscuits

Table 5 and Figure 2 shows the *L*∗, *a*∗, and *b*∗ values of different biscuits blends fortified with banana peel compared with control biscuit prepared from wheat flour. The results observed the significant differences between the colors of control biscuits and those fortified with banana peel flour.

This shows that there was a noticeable color difference in different blends of biscuits fortified with banana peel flour at levels 5, 10, 15, and 20. The change in color may be caused by the extent of Maillard's reaction for the reason that banana peels contain sucrose and protein [36]. Furthermore, enzymes like polyphenol oxidase have been present in the banana peel that may contribute to the brownish color of the flour [37, 38]. [39] noticed that the considerable reduction in the *b*∗ value of the fortified biscuit ranges from 28.08 to 17.38 with partial replacement of wheat flour with amaranth, respectively, at levels of 5, 10, and 15% of substitution.

### 4.7. Texture Profile Analyzer of Biscuits

The texture quality is an important quality feature of biscuits; therefore, the textures of the four best blends of banana peel were tested against that of wheat flour biscuits, and the results are reported in Table 6 and Figure 3.

There were considerably various in the biscuits' texture parameters. This increase was caused by the fiber content of banana peel flour which affects its toughness and other structural features. Mechanical variations referred to the substitute of wheat flour with banana flour in biscuits are associated with an increase in crude fiber, insoluble dietary fiber, fat, and a reduction in carbohydrates. Previous studies [40] found the positive relationship between dietary fibers and hardness and gumminess [41]. In addition, cohesiveness was increased from 0.12 in control biscuits to 0.43 in biscuits made from 20% banana peel flour. This increase might be due to the insoluble dietary fibers from banana peel flour which were substituted for wheat flour.

The results of springiness, gumminess, and chewiness observed that there was a considerably various between the control biscuits and biscuits made from banana peel flour at different levels containing a high amount of insoluble dietary fiber. Moreover, the addition of banana peel flour to the composition of food products does not negatively affect organoleptic attributes such as texture, taste, and smell [42], and it is a low-cost material, rich in insoluble dietary fiber [31].

### 4.8. Effect of Banana Peel on Physical Properties of Biscuits

The physical properties like diameter, high, and spread ratio were determined in control biscuit made from wheat flour with 72% extraction and its blends fortified with banana peel flour at 5, 10, 15, and 20%, and the results in Table 7 and Figure 4 found control biscuit to be significantly higher in physical properties than the other different blends. This means that the noticeable shrinkage in diameter and height can be referred to the dietary fibers, which absorb moisture and help the gluten network to become better by forming an elastic network of the dough which after baking is subject to shrinkage after stretching [43]. These results were confirmed by [44] noticing a decrease in biscuit diameter by adding oven-dried banana peel.

## 5. Conclusion

The study contribution is a banana peel flour containing a high amount of dietary fiber and a rich source of mineral content. These bioactive compounds were used to prepare biscuits as functional foods fortified at levels 5, 10, 15, and 20% from banana peel flour. The color, texture properties, physical analysis, and sensory properties were determined by different blends of biscuits. The different blends prepared from banana peel flour in 5, 10, and 15% levels were acceptable for panelists, while the blend containing 20% banana peel flour was not acceptable and may be caused by dark color and high dietary fiber.

## Figures and Tables

**Figure 1:** Sensory evaluation of biscuits fortified banana peel flour.

**Figure 2:** Color in different blends of biscuit.

**Figure 3:** Texture characteristics of different blends of biscuits.

**Figure 4:** Physical characteristics of different blends of biscuits.

**Table 1:** Nutritional values of banana peel flour on dry weight.

Chemical analysis g/100 g	Banana peel flour	Minerals content mg/100 g	Banana peel flour
Moisture	7.53 ± 0.03	Calcium	80.27 ± 10.16
Protein	6.83 ± 0.02	Phosphorous	217.92 ± 7.04
Ash	9.53 ± 0.05	Iron	42.75 ± 0.11
Fat	4.01 ± .03	Zinc	37.11 ± 1.03
Crude fiber	12.38 ± 0.92	Copper	0.60 ± 0.07
Total carbohydrates	67.25 ± 4.36	Sodium	96.43 ± 3.14
Total dietary fiber	52.68 ± 3.28	Potassium	110.24 ± 6.04
Soluble dietary fiber	10.39 ± 0.86	Magnesium	5.29 ± 0.15
Insoluble dietary fiber	42.29 ± 2.18	Manganese	85.25 ± 4.23

**Table 2:** Nutrition values of biscuits blends (g/100 g dry weight).

Chemical analysis	Control wheat flour	Biscuits blends fortified with banana peel at			
		5%	10%	15%	20%
Moisture	9.12 ± 0.14^a^	9.05 ± 0.17^b^	8.89 ± 0.19^c^	8.65 ± 0.12^d^	8.40 ± 0.12^e^
Protein	10.32 ± 0.28^a^	9.91 ± 0.13^b^	9.51 ± 0.12^c^	9.13 ± 0.13^d^	8.65 ± 0.17^e^
Ash	1.77 ± 0.02^e^	2.36 ± 0.01^d^	2.89 ± 0.05^c^	3.38 ± 0.28^b^	3..93 ± 0.64^a^
Fat	22.05 ± 0.35^e^	22.25 ± 0.42^d^	22.42 ± 0.25^c^	22.61 ± 0.14^b^	22.83 ± 0.19^a^
Crude fiber	1.16 ± 0.04^e^	3.28 ± 0.12^d^	4.47 ± 0.14^c^	5.34 ± 0.17^b^	6.89 ± 0.16^a^
Carbohydrates	64.70 ± 4.03^a^	62.20 ± 4.05^b^	60.71 ± 3.08^c^	59.54 ± 3.07^d^	57.70 ± 2.08^e^
Dietary fiber	3.65 ± 0.08^e^	5.72 ± 0.12^d^	8.22 ± 0.03^c^	11.41 ± 0.02^b^	14.19 ± 0.05^a^
Insoluble dietary fiber	2.54 ± 0.05^e^	3.71 ± 0.14^d^	5.10 ± 0.12^c^	7.30 ± 0.18^b^	9.14 ± 0.13^a^
Soluble dietary fiber	1.21 ± 0.02^e^	2.01 ± 0.18^d^	3.12 ± 0.18^c^	4.11 ± 0.12^b^	5.05 ± 0.15^a^

Each value represents the mean ± SD. Mean followed by different superscript letters in each row are significantly different (*p* < 0.05).

**Table 3:** Minerals content as mg/100 g of biscuits on dry weight.

Minerals content	Control wheat flour	Biscuits fortified with banana peel at			
		5%	10%	15%	20%
Calcium	33.77 ± 1.25^e^	47.25 ± 2.31^d^	61.19 ± 3.58^c^	75.36 ± 4.17^b^	89.35 ± 5.21^a^
Phosphorus	39.34 ± 1.47^c^	42.26 ± 2.68^b^	47.51 ± 2.87^b^	52.17 ± 1.12^b^	57.38 ± 4.59^a^
Iron	2.13 ± 0.05^e^	2.54 ± 0.07^d^	3.14 ± 0.07^c^	3.70 ± 0.09^b^	4.05 ± 0.09^a^
Zinc	1.18 ± 0.08^e^	2.56 ± 0.05^d^	3.62 ± 0.03^c^	4.05 ± 0.07^b^	5.22 ± 0.06^a^
Copper	0.02 ± 0.001^e^	0.32 ± 0.002^d^	0.61 ± 0.07^c^	0.91 ± 0.05^b^	1.21 ± 0.34^a^
Sodium	58.39 ± 2.13^e^	69.33 ± 4..38^d^	71.58 ± 4.18^c^	75.93 ± 3.15^b^	78.33 ± 4.78^a^
Potassium	54.5 ± 2.76^e^	60.11 ± 3.16^d^	66.28 ± 3.73^c^	72.36 ± 3.26^b^	78.29 ± 4.34^a^
Magnesium	4.15 ± 0.03^c^	4.42 ± 0.02^d^	4.92 ± 0.03^c^	5.31 ± 0.04^b^	5.72 ± 0.04^a^
Manganese	15.27 ± 0.77^c^	19.27 ± 0.28^d^	24.12 ± 1.31^c^	29.35 ± 0.95^b^	34.11 ± 1.21^a^

Each value represents the mean ± SD. Mean followed by different superscript letters in each row are significantly different (*p* < 0.05).

**Table 4:** Sensory evaluation of biscuits.

Treatment	Color	Appearance	Flavor	Texture	Taste	Overall
Control	9.00 ± 1.16^a^	9.00 ± 1.33^a^	9.00 ± 0.66^a^	9.00 ± 0.61^a^	9.00 ± 0.87^a^	9.00 ± 0.91^a^
5%	8.25 ± 1.01^b^	8.50 ± 1.13^b^	8.50 ± 0.56^ab^	8.50 ± 0.78^ab^	8.00 ± 0.75^b^	8.35 ± 0.94^b^
10%	7.50 ± 1.19^c^	7.75 ± 1.07^c^	8.25 ± 0.84^ab^	8.00 ± 0.88^b^	7.50 ± 0.75^c^	7.80 ± 0.83^c^
15%	7.00 ± 1.37^d^	7.50 ± 1.07^d^	8.00 ± 0.66^b^	7.50 ± 0.33^c^	7.00 ± 0.58^d^	7.40 ± 0.71^c^
20%	6.25.±1.26^e^	6.75 ± 0.89^e^	7.00 ± 0.71^c^	6.50 ± 0.65^d^	6.00 ± 0.72^e^	6.50 ± 0.52^d^

Each value represents the mean ± SD. Mean followed by different superscript letters in each column are significantly different (*p* < 0.05).

**Table 5:** Color in different blends of biscuits.

Blends of biscuits	*L*∗	*a*∗	*b*∗
Control biscuit	65.14 ± 3.28^a^	4.19 ± 0.03^e^	27.12 ± 0.26^a^
5%	51.35 ± 2.49^b^	7.52 ± 0.06^d^	23.34 ± 0.27^b^
10%	46.42 ± 2.15^c^	11.73 ± 0.13^c^	19.27 ± 0.31^c^
15%	41.18 ± 1.36^d^	15.49 ± 0.17^b^	17.32 ± 0.28^d^
20%	29.67 ± 2.51^e^	19.63 ± 0.21^a^	14.41 ± 0.24^e^

Each value represents the mean ± SD. Mean followed by different superscript letters in each column are significantly different (*p* < 0.05).

**Table 6:** Effect of banana peel on texture characteristics of biscuits.

Treatment	Control	Biscuits fortified with banana peel at			
		5%	10%	15%	20%
Hardness (N)	166.35 ± 7.12^e^	175.46 ± 8.26^d^	205.49 ± 10.10^3c^	240 ± 11.48^b^	295 ± 13.73^a^
Cohesiveness	0.12 ± 0.04^e^	0.19 ± 0.04^d^	0.27 ± 0.10^c^	0.35 ± 0.02^b^	0.43 ± 0.15^a^
Springiness (mm)	1.22 ± 0.07^e^	1.97 ± 0.02^d^	2.67 ± 0.03^c^	3.58 ± 0.09^b^	4.15 ± 0.11^a^
Gumminess(g)	32.28 ± 0.42^e^	40.51 ± 0.65^d^	51.16 ± 0.71^c^	62.18 ± 0.78^b^	70.35 ± 0.86^a^
Chewiness (mJ)	1.43 ± 0, 03^e^	2.27 ± 0.04^d^	2.85 ± 0.05^c^	3.14 ± 0.05^b^	4.71 ± 0.07^a^

Each value represents the mean ± SD. Mean followed by different superscript letters in each row are significantly different (*p* < 0.05).

**Table 7:** Effect of banana peel on physical characteristics of biscuits.

Treatment	Control	Biscuits fortified with banana peel at			
		5%	10%	15%	20%
Diameter (cm)	25.27 ± 0.23^a^	23.97 ± 0.15^b^	22.60 ± 0.17^c^	21.39 ± 0.15^d^	19.76 ± 0.25^e^
High (cm)	7.46 ± 0.07^e^	6.96 ± 0.25^d^	6.25 ± 0.15^c^	5.72 ± 0.12^b^	3.90 ± 0.03^a^
Spread ratio	3.39 ± 0.11^a^	3.44 ± 0.15^b^	3.62 ± 0.03^c^	3.83 ± 0.25^d^	5.07 ± 0.07^e^

Each value represents the mean ± SD. Mean followed by different superscript letters in each row are significantly different (*p* < 0.05).

## Data Availability

The data used to support the findings of this study are included within the article.
